The article "DNA barcoding detects contamination and substitution in North American herbal products" was retracted in 2024. Reason: fabricated or falsified data.

# DNA barcoding detects contamination and substitution in North American herbal products

**DOI:** 10.1186/1741-7015-11-222

**Published:** 2013-10-11

**Authors:** Steven G Newmaster, Meghan Grguric, Dhivya Shanmughanandhan, Sathishkumar Ramalingam, Subramanyam Ragupathy

**Affiliations:** 1 Centre for Biodiversity Genomics, Biodiversity Institute of Ontario (BIO), University of Guelph, Guelph, Ontario N1G 2W1, Canada; 2 Bachelor of Arts and Science Program, University of Guelph, Guelph, Ontario N1G 2W1, Canada; 3 Plant Genetic Engineering Laboratory, Department of Biotechnology, Bharathiar University, Coimbatore 641 046, Tamil Nadu, India

## Abstract

**Background:**

Herbal products available to consumers in the marketplace may be contaminated or substituted with alternative plant species and fillers that are not listed on the labels. According to the World Health Organization, the adulteration of herbal products is a threat to consumer safety. Our research aimed to investigate herbal product integrity and authenticity with the goal of protecting consumers from health risks associated with product substitution and contamination.

**Methods:**

We used DNA barcoding to conduct a blind test of the authenticity for (i) 44 herbal products representing 12 companies and 30 different species of herbs, and (ii) 50 leaf samples collected from 42 herbal species. Our laboratory also assembled the first standard reference material (SRM) herbal barcode library from 100 herbal species of known provenance that were used to identify the unknown herbal products and leaf samples.

**Results:**

We recovered DNA barcodes from most herbal products (91%) and all leaf samples (100%), with 95% species resolution using a tiered approach (*rbcL* + *ITS2*). Most (59%) of the products tested contained DNA barcodes from plant species not listed on the labels. Although we were able to authenticate almost half (48%) of the products, one-third of these also contained contaminants and or fillers not listed on the label. Product substitution occurred in 30/44 of the products tested and only 2/12 companies had products without any substitution, contamination or fillers. Some of the contaminants we found pose serious health risks to consumers.

**Conclusions:**

Most of the herbal products tested were of poor quality, including considerable product substitution, contamination and use of fillers. These activities dilute the effectiveness of otherwise useful remedies, lowering the perceived value of all related products because of a lack of consumer confidence in them. We suggest that the herbal industry should embrace DNA barcoding for authenticating herbal products through testing of raw materials used in manufacturing products. The use of an SRM DNA herbal barcode library for testing bulk materials could provide a method for 'best practices? in the manufacturing of herbal products. This would provide consumers with safe, high quality herbal products.

## Background

Globalization of trade is expanding natural product commodity markets that sustain life and promote good health, yet the challenging financial climate is squeezing profit margins and exacerbating the propensity for contamination, fraudulent market substitution and the use of unlabeled fillers. This comes at a time when consumers are becoming increasingly concerned about the authenticity of the products they purchase. North America is a major provider of goods such as herbal products, a commodity that has come under scrutiny recently in the media due to product substitution [1-3].

The International Trade in herbal products is a major force in the global economy and the demand is increasing in both developing and developed nations. There are currently more than 1,000 companies producing medicinal plant products with annual revenues in excess of US$60 billion. Notably, medicinal herbs now constitute the most rapidly growing segment of the North American alternative medicine market [4,5], with over 29,000 herbal substances [6,7] generating billions of dollars in trade. These statistics are indicative of the rapid growth (>15%/year) in the marketplace for natural plant products and the broadening consumer base interested in herbal products from India, Canada, USA and Europe. Yet, as highlighted in recent media reports, product adulteration and ingredient substitution is not uncommon as species of a lower market value are substituted for those of a higher value. This practice constitutes not only product fraud, but according to the World Health Organization (WHO), the adulteration of herbal products is a threat to consumer safety (see Discussion). Eroding consumer confidence is driving the demand for research and market testing on herbal product authentication.

There are currently no best practices in place for identifying the species of the various ingredients used in herbal products. This is because the diagnostic morphological features of the plants on which the current Linnaean taxonomic system is based cannot typically be assessed from powdered or otherwise processed biomaterials. As a result, the marketplace is prone to contamination and possible product substitution, which dilute the effectiveness of otherwise useful remedies, lowering the perceived value of all related products because of a lack of consumer confidence in them. Herbal product substitution has been documented for many individual medicinal plant species [8-10], teas [1] and 'nutraceuticals? [11,12]. Although there is limited research available, the frequency of product mislabeling in herbal products has been estimated at 14% to 33% from previous studies [1-3]. There are legitimate health concerns for consumers which results in a lack of confidence in safe, high quality herbal products.

A broadly accessible commercial tool to detect product substitution and develop best practices for authentication of many commercial products is beginning to emerge. DNA barcoding has been used to test a number of natural products [1,3,13]. Barcoding uses state-of-the-art biotechnology to help identify plant material based on short, standardized gene sequences, in a rapid, accurate and cost-effective manner. For example, Srirama *et al.*[10] has demonstrated the efficiency of DNA barcoding in identifying adulterants in the raw drug trade of *Phyllanthus* (Euphorbiaceae). *Phyllanthus* is one of the most important groups of species traded as a raw herbal drug treatment for liver disorders [14]. This study showed that plant DNA barcoding can effectively discriminate *Phyllanthus* species, and hence can be used to resolve species admixtures in the raw drug trade samples; there are several phenotypically similar species that could easily be misidentified and mixed within herbal products. Over the last 3 years, studies of Chinese plant medicine [15-20] have documented the potential scope and magnitude of market substitution using this biotechnology. However, there are only a few studies [1,3] available, and they provide a limited assessment of the authenticity of commercial herbal products within the marketplace. Currently there is a gap in our understanding to the extent of herbal product substitution, contamination and use of fillers. Also, there are no studies that have used a standard reference material (SRM) herbal barcode library and barcode regions that facilitate species resolution.

This study utilized blind sampling of commercially available herbal products, which were tested for authentication of plant ingredients using an SRM herbal DNA barcode library. Our research questions focused on the following three areas. (1) Authentication: is the herbal species on the label found in the product? (2) Substitution: is the main herbal ingredient substituted by other species? (3) Fillers: are there any unlabeled fillers used?

## Methods

### Study design

We tested the authenticity of 44 (41 capsules; 2 powders; 1 tablet) herbal products representing 12 companies. The samples were submitted in a blind test for authentication (product no. label only) using DNA barcoding at the Centre for Biodiversity Genomics (CBG) within the Biodiversity Institute of Ontario (BIO), University of Guelph.

The project also included a second blind test in which we barcoded 50 leaf samples (blind labels) collected from living samples of known provenance from horticultural greenhouses. These leaf samples represented 42 species including all those listed on the herbal product labels and some closely related species. This provided an independent test of the ability of barcoding to differentiate all the species on the herbal product labels used in this study. All of the samples are in the Barcode of Life Database (BOLD) (Additional file 1: Table S1) and GenBank (Additional file 2: Table S2). All vouchers are scanned and recorded in the BOLD and deposited in the BIO Herbarium at the University of Guelph.

### Herbal product sampling

In North America, herbal products are available in a variety of mainstream outlets such as supermarkets, health food stores, pharmacies and can be ordered online from herbal supply companies. In our study, samples were collected in the greater Toronto area (GTA) in Canada, with several samples mailed from distributors in the USA. All products are available to consumers in both Canada and the USA. The herbal product samples represented 30 herbal species that were each represented by 2 or 3 different companies.

### DNA barcoding (DNA extraction and sequencing)

We barcoded triplicate samples of plant product (powder) from the 44 herbal products and 50 herbal leaf samples using a tiered approach (*rbcL* + *ITS2*) [21]. Multiple DNA extracts (five to ten) were taken from each of these triplicate samples of which these DNA extracts were barcoded to make sure we did not miss any species? DNA. Since these were only single ingredient herbal products we did not expect to detect more than one plant species barcode unless it was a contaminant. However, our intensive DNA extract sampling allowed us to sample for other plant polymerase chain reaction (PCR) products, which were then sequenced separately. This included building barcode sample by species curves to see how many times we needed to sample to get an accurate estimate of species in a sample. As a result some of the products yielded two difference sequences, each from DNA extracts taken from the same sample product.

Total genomic DNA was isolated from 100 mg of the dry material using the Nucleospin Plant II Mini DNA Extraction kit. The PCR amplification was performed in a 20 ?L reaction mixture that contained 2.5 ?L of genomic DNA, 2.5 ?L of 10 ? *Pfu* buffer with MgSO_4_ (Fermentas?), 2.5 ?L of 2 mM dNTPs (Fermentas), 0.5 ?L each of forward and reverse primers (10 pM) and 0.2 ?L of 2.5 U *Pfu* DNA Polymerase (Fermentas) and 2 ?L 0.5% dimethylsulfoxide (DMSO). The primers and the reaction conditions are previously published for *rbcL*[22] and *ITS*2 [16]. Touchdown PCR was carried out. The PCR products obtained from these reactions were subjected to Big Dye (version 3.1) sequencing reactions that had a total volume of 10 ?L and included 10 pMol of each primer. The sequencing amplification protocol consisted of 1 cycle of 1 minute at 96?C, followed by 30 cycles of 10 s at 96?C, 5 s at 55?C, and 4 minutes at 60?C. The amplicons were bidirectionally sequenced using ABI 377 sequencer (Applied Biosystems). The chromatographic traces were aligned and codon read in the Codoncode Aligner ver. 3.0 (CodonCode, Dedham, MA, USA) and contigs were generated. Sequences were deposited in BOLD and GenBank.

### SRM herbal barcode library

An SRM herbal barcode library was prepared and used to identify the unknown herbal products and leaf samples. This library was assembled from 100 herbal species of known provenance that were identified by taxonomic experts. These samples were prepared into herbarium vouchers and are archived at the BIO Herbarium and in the BOLD. Although our library contained 100 herbal species in this study it is part of a larger project in which we are currently expanding the SRM herbal barcode library to include the main species used within herbal product industry in North America.

### Product identification and analysis

Identification of unknown barcodes from products and leaves was conducted by comparing Basic Local Alignment Search Tool (BLAST) data against our SRM herbal barcode library with a minimum BLAST cut off of 97% identity for a top match [3]. These results were verified by neighbor-joining tree analysis in which we compared the branches of unknown specimens to sequences of reference species. A species is considered as taxonomically resolved if its members showed at least one diagnostic difference from any other taxon in the study and formed a monophyletic clade.

The definitions of terms used when assessing the identity of DNA barcodes recovered from herbal products are as outlined below.

#### Authentic

A product is authentic if it contains a DNA barcode for a species that is the main ingredient on the label of a tested herbal product.

#### Contamination

A product is contaminated if a DNA barcode is found for a species other than what is labeled on the tested product, in addition to the authentic barcode; this could include known herbal product filler species (see below).

#### Substitution

Product substitution occurs when a DNA barcode is found for a species other than what is labeled on the tested product, AND there is NOT a barcode recovered for the main ingredient listed. Note that this strict definition does not consider whether it is an accidental misidentification of a bulk product or a fraudulent market substitution for a cheaper product.

#### Filler

A product contains fillers if a DNA barcode is found for known herbal product filler species including rice (*Oryza sativa*), soybean (*Glycine max*) and wheat (*Triticum* spp.). Fillers may be found in place of (substitution) or in addition to the barcode of the main product ingredient (contamination).

## Results

### DNA barcode success

Recovery of DNA barcodes from various herbal products was successful. High quality DNA barcodes were obtainable for both *rbcL* and *ITS2* regions for 100% of the 100 vouchered herbal species (Ontario Agricultural College Herbarium), which served as a high quality SRM herbal barcode library. This library provided a database that could be used to identify unknown haplotypes (barcodes) recovered from herbal products. The SRM classification tree (Figure? 1) shows that all herbal species have 100% species resolution, with each species presenting at least one diagnostic difference from any other taxon and formed a monophyletic clade (Figure? 1). Herbal product DNA barcode success rate was 91% (40/44 products) for the combined regions, resulting in the recovery of 34 *rbcL* and 40 *ITS2* sequences. Species resolution for barcodes recovered from herbal products was 66% (*rbcL*) and 93% (*ITS2*). Low resolution in *rbcL* was expected, because it is known to have insufficient nucleotide sequence variability to distinguish among closely related species. The three unresolved species with *ITS2* was due to three samples that had product substitution with species that were not in our SRM library; these unknown species barcodes did match the nearest family and genus. We also barcoded blindly labeled herbal leaf samples collected from living samples from horticultural greenhouses. This provided an independent test of the ability of barcoding to differentiate all the species on the herbal product labels. Species resolution for barcodes recovered from the herbal leaf samples was 57% (*rbcL*) and 100% (*ITS2*), with perfect matches to the herbal SRM barcode library using BLAST.

**Figure 1:** **Standard reference material (SRM) herbal barcode library consensus tree (MP-ratchet analysis) for combined barcode data from *rbc L*and *ITS2 *from 100 herbal species of known provenance that were identified by taxonomic experts.**

### Authentication: is the herbal species on the label found in the product?

What is listed on the label of herbal products is not always what is found within the product. DNA barcoding was able to authenticate 48% of the products tested (Figure? 2). However, most (59%) of the herbal products tested contained species of plants not listed on the labels (Figure? 2). Some (33%) of the authenticated herbal products also contained contaminants and or fillers not listed on the label (Figure? 2). Some of the DNA sequences recovered were only identified to family as our SRM herbal DNA barcode library is not yet complete (see note above). However, an incomplete SRM barcode library still allows a correct identity in a hierarchical way to family and genera depending on the level of best match within the classification tree. Some of the contaminants were of unrelated species from entirely different plant families (Table? 1). Although many of the herbal companies (75%) whose product we tested did have some authentic products, only 2 of the 12 companies provided authentic products with no substitution, contaminants or fillers. Conversely, we were unable to authenticate any of the products for 25% of the companies (Figure? 3). Although these numbers shed light on the number of companies with authenticate products we only sampled three or four products per company and therefore differences among companies are likely due to chance.

**Figure 2:** DNA barcode results from blind testing of the 44 herbal products representing 30 medicinal species of plants.

**Table 1:** DNA barcode results listed for individual samples from blind testing of the 44 herbal products and 50 herbal leaf samples representing 42 medicinal species of plants

**Market label or Herb leaf species**	**Sample from**	**Barcode ID**	**ITS2 ID**	**rbcL ID**
*Achillea millefolium* (Yarrow)	HP64C	*Achillea millefolium + Medicago sativa*^a^	*Achillea millefolium + Medicago sativa*^a^	*Medicago sativa*^a^
*Achillea millefolium*	HP56L	*Achillea millefolium*	*Achillea millefolium*	*Achillea sp.*
*Actaea racemosa* (Cohosh)	HP42C	*Actaea asiatica*^a^	*Actaea asiatica*^a^	*Actaea asiatica*^a^
*Actaea racemosa*	HP20C	NS	NS	NS
*Actaea racemosa*	HP45L	*Actaea racemosa*	*Actaea racemosa*	*Actaea racemosa*
*Actaea racemosa*	HP74L	*Actaea racemosa*	*Actaea racemosa*	*Actaea racemosa*
*Actaea racemosa*	HP77L	*Actaea racemosa*	*Actaea racemosa*	*Actaea racemosa*
*Amaranthus sp.* (Amaranth)	HP89P	*Amaranthus sp.*	*Amaranthus sp.*	*Amaranthus sp.*
*Amaranthus albus*	HP79L	*Amaranthus albus*	*Amaranthus albus*	*Amaranthus sp.*
*Amaranthus retroflexus*	HP49L	*Amaranthus retroflexus*	*Amaranthus retroflexus*	*Amaranthus sp.*
*Apium graveolens* (Celery)	HP34C	*Amaryllidaceae + Oryza sativa*^a^	*Amaryllidaceae*^a^	*Oryza sativa*^b^
*Apium graveolens*	HP32C	NS	NS	NS
*Apium graveolens*	HP43C	NS	NS	NS
*Apium graveolens*	HP13L	*Apium graveolens*	*Apium graveolens*	*Apiaceae*
*Apium graveolens*	HP5L	*Apium graveolens*	*Apium graveolens*	*Apiaceae*
*Apium graveolens*	HP51L	*Apium graveolens*	*Apium graveolens*	*Apiaceae*
*Arctium lappa* (Burdock)	HP6C	*Arctium lappa*	*Arctium lappa*	*Arctium lappa*
*Arctium lappa*	HP22C	*Oryza sativa*^a^	*Oryza sativa*^b^	*Oryza sativa*^b^
*Arctium lappa*	HP21C	*Ranunculaceae*^a^	*Ranunculaceae*^a^	NS
*Arctium lappa*	HP4L	*Arctium lappa*	*Arctium lappa*	*Arctium lappa*
*Arctium lappa*	HP92L	*Arctium lappa*	*Arctium lappa*	*Arctium lappa*
*Cinnamomum cassia (Cinnamon)*	HP86T	*Ranunculaceae*^a^	*Ranunculaceae*^a^	NS
*Cinnamomum cassia (Cinnamon)*	HP60L	*Cinnamomum cassia*	*Cinnamomum cassia*	*Cinnamomum sp.*
*Echinacaea purpurea* (Echinacaea)	HP35C	*Echinacaea purpurea + Parthenium hysterophorus*^a^	*Echinacaea purpurea + Parthenium hysterophorus*^a^	*Asteraceae*^a^
*Echinacaea purpurea*	HP27C	*Echinacaea purpurea + Parthenium hysterophorus*^a^	*Echinacaea purpurea + Parthenium hysterophorus*^a^	*Asteraceae*^a^
*Echinacaea purpurea*	HP88L	*Echinacaea purpurea*	*Echinacaea purpurea*	*Echinacaea purpurea*
*Echinacaea purpurea*	HP80L	*Echinacaea purpurea*	*Echinacaea purpurea*	*Echinacaea purpurea*
*Echinacaea purpurea*	HP70L	*Echinacaea purpurea*	*Echinacaea purpurea*	*Echinacaea purpurea*
*Echinacaea purpurea*	HP85L	*Echinacaea purpurea*	*Echinacaea purpurea*	*Echinacaea purpurea*
*Ginkgo biloba* (Ginkgo)	HP63C	*Ginkgo biloba*	*Ginkgo biloba*	*Ginkgo biloba*
*Ginkgo biloba*	HP28C	*Juglans nigra*^a^	*Juglans nigra*^a^	NS*
*Ginkgo biloba*	HP81C	*Oryza sativa*^a^	*Oryza sativa*^b^	*Oryza sativa*^b^
*Ginkgo biloba*	HP33L	*Ginkgo biloba*	*Ginkgo biloba*	*Ginkgo biloba*
*Ginkgo biloba*	HP2L	*Ginkgo biloba*	*Ginkgo biloba*	*Ginkgo biloba*
*Ginkgo biloba*	HP78L	*Ginkgo biloba*	*Ginkgo biloba*	*Ginkgo biloba*
*Ginkgo biloba*	HP16L	*Ginkgo biloba*	*Ginkgo biloba*	*Ginkgo biloba*
*Hypericum perforatum* (St. John?s wort)	HP8C	*Fabaceae*^a^	*Fabaceae*^a^	NS
*Hypericum perforatum*	HP46C	*Hypericum perforatum*	*Hypericum perforatum*	*Hypericum perforatum*
*Hypericum perforatum*	HP82C	*Oryza sativa*^a^	*Oryza sativa*^b^	*Oryza sativa*^b^
*Hypericum perforatum*	HP39L	*Hypericum perforatum*	*Hypericum perforatum*	*Hypericum perforatum*
*Hypericum perforatum*	HP94L	*Hypericum perforatum*	*Hypericum perforatum*	*Hypericum perforatum*
*Juglans nigra* (Walnut)	HP40C	*Juglans nigra*	*Juglans nigra*	NS
*Juglans nigra*	HP58C	NS	NS	NS
*Juglans nigra*	HP84C	*Oryza sativa*^a^	NS	*Oryza sativa*^b^
*Juglans nigra*	HP30L	*Juglans nigra*	*Juglans nigra*	*Juglans nigra*
*Juglans nigra*	HP19L	*Juglans nigra*	*Juglans nigra*	*Juglans nigra*
*Juglans nigra*	HP17L	*Juglans nigra*	*Juglans nigra*	*Juglans nigra*
*Matricaria recutita (Chamomile)*	HP37C	*Matricaria recutita*	*Matricaria recutita*	*Matricaria recutita*
*Matricaria recutita (Chamomile)*	HP91C	*Matricaria recutita + Medicago sativa*	*Matricaria recutita + Medicago sativa*	*Medicago sativa*
*Matricaria recutita (Chamomile)*	HP36C	*Matricaria recutita + Glycine max*	*Matricaria recutita*	*Glycine max*
*Matricaria recutita*	HP76L	*Matricaria recutita*	*Matricaria recutita*	*Matricaria recutita*
*Mentha arvensis* (Mint)	HP3C	*Mentha arvensis*	*Mentha arvensis*	*Lamiaceae*
*Mentha arvensis*	HP52L	*Mentha arvensis*	*Mentha arvensis*	*Lamiaceae*
*Mentha spicata*	HP15L	*Mentha spicata*	*Mentha spicata*	*Lamiaceae*
*Nepeta cataria*	HP9L	*Nepeta cataria*	*Nepeta cataria*	*Lamiaceae*
*Oenothera biennis* (Evening Primrose)	HP48C	*Oenothera biennis*	*Oenothera biennis*	*Oenothera biennis*
*Origanum vulgare* (Oregano)	HP10C	*Origanum vulgare + Lamiaceae*^a^	*Origanum vulgare + Lamiaceae*^a^	*Lamiaceae*^a^
*Oenothera biennis*	HP47L	*Oenothera biennis*	*Oenothera biennis*	*Oenothera biennis*
*Origanum vulgare*	HP26L	*Origanum vulgare*	*Origanum vulgare*	*Origanum vulgare*
*Origanum vulgare*	HP50L	*Origanum vulgare*	*Origanum vulgare*	*Origanum vulgare*
*Oxalis Corniculata* (WoodSorrel)	HP1P	*Oxalis Corniculata + Medicago sativa*^a^	*Oxalis Corniculata + Medicago sativa*^a^	*Oxalis sp.*
*Oxalis Corniculata*	HP72L	*Oxalis Corniculata*	*Oxalis Corniculata*	*Oxalis sp.*
*Oxalis stricta*	HP57L	*Oxalis stricta*	*Oxalis stricta*	*Oxalis sp.*
*Oxalis acetosella*	HP18L	*Oxalis acetosella*	*Oxalis acetosella*	*Oxalis sp.*
*Plantago ovate* (Psyllium)	HP69C	*Plantago ovate*	*Plantago ovate*	NS
*Plantago ovate*	HP71L	*Plantago ovate*	*Plantago ovate*	*Plantago sp.*
*Plantago major*	HP66L	*Plantago major*	*Plantago major*	*Plantago sp.*
*Plantago lanceolata*	HP14L	*Plantago lanceolata*	*Plantago lanceolata*	*Plantago sp.*
*Portulaca oleracea* (Purslane)	HP83C	*Portulaca oleracea*	*Portulaca oleracea*	*Portulaca oleracea*
*Portulaca oleracea*	HP65C	*Portulaca oleracea + Glycine max*^b^	*Portulaca oleracea + Glycine max*^b^	*Glycine max*^b^
*Portulaca oleracea*	HP38L	*Portulaca oleracea*	*Portulaca oleracea*	*Portulaca oleracea*
*Portulaca oleracea*	HP93L	*Portulaca oleracea*	*Portulaca oleracea*	*Portulaca oleracea*
*Rubus idaeus* (Raspberry)	HP24C	*Rubus idaeus*	*Rubus idaeus*	*Rubus sp.*
*Rubus idaeus*	HP12C	*Rubus idaeus + Medicago sativa*^a^	*Rubus idaeus + Medicago sativa*^a^	*Medicago sativa*^a^
*Rubus idaeus*	HP61L	*Rubus idaeus*	*Rubus idaeus*	*Rubus sp.*
*Rubus parviflorus*	HP29L	*Rubus parviflorus*	*Rubus parviflorus*	*Rubus sp.*
*Rudbeckia hirta* (black-eyed Susan)	HP62C	*Rudbeckia hirta*	*Rudbeckia hirta*	*Rudbeckia hirta*
*Rudbeckia hirta*	HP31L	*Rudbeckia hirta*	*Rudbeckia hirta*	*Rudbeckia hirta*
*Sambucus nigra (Elderberry)*	HP23C	*Sambucus nigra + Medicago sativa*^a^	*Sambucus nigra + Medicago sativa*^a^	*Sambucus sp.*
*Sambucus nigra*	HP59L	*Sambucus nigra*	*Sambucus nigra*	*Sambucus sp.*
*Sambucus racemosa*	HP54L	*Sambucus racemosa*	*Sambucus racemosa*	*Sambucus sp.*
*Sonchus arvensis* (Thistle)	HP87C	*Sonchus arvensis*	*Sonchus arvensis*	*Sonchus arvensis*
*Sonchus arvensis*	HP67C	*Sonchus arvensis + Medicago sativa*^a^	*Sonchus arvensis + Medicago sativa*^a^	*Sonchus arvensis*
*Sonchus arvensis*	HP73L	*Sonchus arvensis*	*Sonchus arvensis*	*Sonchus arvensis*
*Sonchus asper*	HP41L	*Sonchus asper*	*Sonchus asper*	*Sonchus asper*
*Symphytum officinale* (Comfrey)	HP7C	*Symphytum officinale + Medicago sativa*^a^	*Symphytum officinale + Medicago sativa*^a^	*Medicago sativa*^a^
*Symphytum officinale*	HP90L	*Symphytum officinale*	*Symphytum officinale*	*Boraginaceae*
*Taraxacum officinale*	HP25C	*Parthenium hysterophorus*^a^	*Parthenium hysterophorus*^a^	*Asteraceae*^a^
*Taraxacum officinale*	HP11C	*Taraxacum officinale + Panicum sp.*^a^	*Taraxacum officinale + Panicum sp.*^a^	*Panicum sp.*^a^
*Taraxacum officinale*	HP75C	*Triticum spp. + Musa sp.*^a^	*Triticum spp. + Musa sp.*^a^	*Musaceae*^a^
*Taraxacum officinale*	HP53L	*Taraxacum officinale*	*Taraxacum officinale*	*Taraxacum officinale*
*Urtica dioica* (Nettles)	HP55C	*Urtica dioica*	*Urtica dioica*	*Urtica dioica*
*Urtica dioica*	HP44C	*Urtica dioica + Oryza sativa*^b^	*Urtica dioica*^b^	*Oryza sativa*^b^
*Urtica dioica*	HP68L	*Urtica dioica*	*Urtica dioica*	*Urtica dioica*

^a^Designates product contamination or substitution.

^b^Refers to use of fillers.

*C* capsule, *L* leaf, *NS* no sequence, *P* powder, *T* tablet.

**Figure 3:** DNA barcode results from blind testing of the 44 herbal products representing 12 companies.

### Substitution: is the main herbal ingredient substituted for some other species?

Our barcoding analysis of 44 herbal products representing 30 medicinal plants species identified product substitution in 32% of the samples (Figure? 2; Table? 1). The criteria we used to determine product substitution was the identity of other plant taxa in place of the product?s main labeled ingredient, which was NOT detected within the sample. We detected product substitution within most (83%) of the 12 companies that we tested (Figure? 3). It should be noted that for 90% of the herbal species in this study, there were product(s) from at least one company that yielded a correct identity (indicating an authentic product). This is confirmation that processing is not an impediment to recovering barcodes. It should also be noted that we sampled each product intensively without replacement; multiple samples per product were extracted and barcoded to make sure we did not miss any species? DNA. Since these were only single ingredient herbal products we did not expect to detect more than one plant species barcode unless it was a contaminant. Our intensive sampling yielded a maximum of two species barcodes per herbal product of which one was either the correct herbal product species or a substitute, and the other was either a filler or contaminant.

### Fillers: are there unlabeled fillers used in herbal products?

Some of the herbal products contained fillers that were not listed on the labels. Our definition is limited to the detection of DNA barcodes from *O. sativa* and *G. max*. These filler species were detected within 21% of the products. We also detected grasses in the samples, which also included wheat (*Triticum* spp.). It is not known whether or not these plants were intentionally used as fillers or if they are contaminants; we are currently investigating the use of fillers in processing by each individual company. In 9% of the samples only rice or wheat barcodes were detected; there were no barcodes detected for the herbal species on the label. The use of fillers was limited to one-third of companies whose products we tested (Figure? 3).

## Discussion

### Contamination and substitution in North American herbal products

Few studies have attempted to estimate how prevalent herbal product contamination and substitution is in the marketplace. To date there are only a few [1-3] studies of herbal product substitution, representing <1% of the herbal products and <5% of the herbal companies in North America. These studies document species-level DNA barcode identification success for 42% to 66% of the herbal species tested. Our study demonstrates increased testing and success, including (i) species-level DNA barcode identification success to 95% of the herbal species tested, and (ii) herbal market testing by approximately 20% for both products and companies. Although we provide new estimates of herbal product contamination and substitution, we caution that these values need to be refined by further studies as we have yet to sample >1% market. However, our estimates do corroborate those of other studies. For example, Stoeckle *et al.*[1] investigated contamination in 131 herbal tea products representing 48 herbal species and found that although they were able to authenticate 58% of the products, 33% of the herbal teas tested were contaminated. Similar estimates from a marketplace survey [2] of 40 dietary supplement products labeled as 'black cohosh? (*Actaea racemosa*) found that 75% of the samples were authentic black cohosh, whereas 25% were substituted with 4 closely related Asian *Actaea* species (*A. asiatica*, *A. cimicifuga*, *A. dahurica*, and *A. simplex*). We also found substitution of black cohosh for Asian *Actaea*, as did another study by Wallace *et al.*[3]. Wallace *et al.*[3] also documented that 50% of ginseng products labeled 'Korean ginseng (*Panax ginseng*)? were actually American ginseng (*Panax quinquefolius*). Although the DNA barcode success rate was low (48%, see below) in Wallace?s study, they were still able to detect product substitution in 14% of the herbal samples tested, representing 7 species of herbs in 14 products. This study also detected fillers in 21% of the herbal products [3]. We found alfalfa (*Medicago sativa*) in 16% of the products tested, which was also previously detected in teas [1]. It is unlikely that this was a contaminant as it was found in so many of the products in addition to the main ingredient. It may be possible that this species is used by some companies as a cheap filler as it is commonly grown and bailed in agricultural areas, and available in large quantities throughout the year.

Contamination and substitution in herbal products present considerable health risks for consumers. In our study, we found contamination in several products with plants that have known toxicity, side effects and/or negatively interact with other herbs, supplements, or medications. For example, we found that one product (HP8) labeled as St. John?s wort (*Hypericum perforatum*) was substituted with *Senna alexandrina* (fabaceae); it contained only senna barcodes and no St. John?s wort barcodes. This is a serious health risk as senna is a Food and Drug Administration (FDA)-approved non-prescription herbal laxative, which is not for prolonged use as it can cause adverse effects such as chronic diarrhea, cathartic colon, liver damage, abdominal pain, epidermal breakdown and blistering [23,24]. Senna contains several unique glycosides called sennosides that interact with immune cells in the colon [25]. We also found contamination of several herbal products (Table? 1) with *Parthenium hysterophorus* (feverfew)*.* Feverfew is native to Eurasia and is an invasive weed in Europe, the Mediterranean, North America and Chile. Although feverfew has been used to treat fever, migraine headaches and arthritis, it does have negative side effects such as swelling and numbness of the mouth, oral ulcers, nausea, vomiting, abdominal pain, diarrhea, and flatulence; some users experienced withdrawal syndromes when discontinuing use, such as rebound headaches and muscle and joint pain [26,27]. Feverfew reacts with a variety of medications metabolized by the liver and may also increase the risk of bleeding, especially if taken with blood-thinning medications such as warfarin or aspirin [28,29]. Pregnant women should not consume any amount of feverfew [29]. Feverfew can also cause allergic reactions, including contact dermatitis due to a toxin found in this plant species called parthenin [30,31]. Although it is not known how contamination with feverfew occurred in this product, it is possible that it was a common weed in the crop used to make this herbal product.

We also found contamination of a Ginkgo product with *Juglans nigra* (black walnut). Wallace *et al.*[3] also found contamination of an *Echinacea* product with walnut and advised that such contamination would be particularly dangerous for a consumer with nut allergies. However, we feel it is unlikely that nuts are the source of contamination, but rather leaves that often litter a very large area surrounding a tree in mid to late summer. It is conceivable that there may have been a field of commercial herbs bordered by walnuts (a common occurrence on the landscape), and that the target crop was harvested along with walnut leaves. Walnut leaves, woods, bark and fruits all contain juglone [32], which is toxic; juglone can lead to oxidative stress or electrophilicity [33-35]. The Registry of Toxic Effects of Chemical Substances (RTECS?) [36] defines juglone as an equivocal tumorigenic agent (lungs, thorax and respiration, skin and appendages), which has been shown to promote skin tumors [37-39]. Ours and other studies [1,3] of herbal product contamination in the marketplace have not been able to identify all the contaminants to species-level resolution due to the lack of a complete SRM barcode library for herbal plants; a complete SRM library would include herbal species, related species and known toxic plants. It is possible that there were other contaminants that were missed because they could only be identified to family rather than to species.

Unlabeled plant fillers may also be found in herbal products, and these fillers are in some cases a potential health risk for consumers. DNA barcoding in our study identified several potential fillers, including rice (*O. sativa*), soybean (*G. max*) and various grasses such as wheat (*Triticum* spp.). This is a health concern for people allergic to these plants, as well as for people seeking gluten free products. Wallace *et al.*[3] found rice and soybean fillers in natural plant and animal products and suggested that these fillers may produce a mixed signal during the sequencing process, contributing to a rather high percentage of failed sequencing reactions in capsulated products. We did not share this high percentage of sequence failures and found barcodes from both the herbal species on the label and fillers within the same product, suggesting that there may be fillers substituted for authentic herbal species. It is probable that barcoding detected rice and soybean, which is a common microcrystalline cellulose and gelatin used as additives in preparing the capsules that contain the herbal product [40]. It is also common practice in the natural products industry to use fillers such as those listed above, which are mixed with the active ingredients. Nonetheless, the consumer has a right to see all of the plant species used in producing a natural product on the list of ingredients.

### Challenges and biotechnical advances in DNA barcoding of herbal products

Authentication of herbal products is challenging, but new DNA barcoding methods are providing tools for routine market analysis [41]. Several major challenges include the lack of an SRM herbal barcode library, and use of only plastid barcode regions, which has resulted in low species resolution. The original definition of a reliable DNA identification of species requires (i) recovery of a barcode sequence from the sample, (ii) representation of relevant species in the reference database, and (iii) sufficient nucleotide sequence variability to distinguish among closely related species [42]. We are designing new protocols for recovering DNA barcodes from herbal samples, which satisfies the first requirement, but the second requirement of a reference database has yet to be satisfied. This problem has been discussed in previous market studies that have tested the authenticity of herbal products without a herbal SRM barcode library [1-3]. These studies have defined the uncertainties of assigning unknown haplotypes from herbal products using incomplete reference barcode databases in GenBank and BOLD. The use of GenBank is inappropriate given that many of the DNA sequences do not have vouchers to professionally identified specimens archived in a herbarium. Therefore the reference sequence in GenBank may be from an incorrectly identified plant and there is no way to verify the specific origin of that DNA. Similarly, the 'Medicinal Materials DNA Barcode Database? [43] provides barcodes for many species of medicinal plants for which there is no record of vouchers to confirm identity; this is an essential component of any DNA Barcode [42]. Our study is the first to build a partial herbal SRM barcode library using vouchered samples of known provenance that was used to test the identity of unknown barcodes recovered from herbal products. Although we only have 100 species in the SRM library, we expect to expand this to over 200 species by the end of 2013, and 1,000 species by 2015. However, this will only add up to 55% of the 1,800 medicinal plant species that are commercially available [44]. If we want to have reliable identifications using DNA barcodes we must build an SRM herbal barcode library that has all sister species for the 1,800 known medicinal species used in commercial products. This is one of the goals of our Herb-BOL (barcode of life) research program in the next 5 years.

The use of only plastid barcode regions is problematic for testing herbal products. Previous studies have not satisfied Hebert?s third criteria for a reliable barcode: sufficient nucleotide sequence variability to distinguish among closely related species [42]. Other studies have adopted the core plant barcodes of *rbcL*a and *matK* genes [45]. We do not recommend using *matK* because of associated problems we encountered with PCR amplification while working on nutmeg [46]. Other published studies have also encountered similar problems [47-51]. We recommend a tiered [21] approach to analysis as one way to overcome the issue of alignment with non-coding regions, while providing the most variability from two-barcode regions for identifying closely related taxa. The tiered approach is based on the use of a common, easily amplified, and aligned region such as *rbcL* that can act as a scaffold on which to place data from a highly variable region such as *ITS2*. The use of *rbcL* as a primary tier barcode is appropriate because of its universality, ease of amplification, ease of alignment, and because there is a significant body of data available for evaluation [51,52]. We prefer to use *ITS2* as the second tier as proposed by Chen *et al.*[16] for use in identifying medicinal plants because (i) it provides high species resolution, (ii) it is from the nuclear genome, which evolves at a different rate than the plastid genome, and (iii) it is a much shorter sequence allowing higher recovery from processed plant materials found within herbal products. The use of *rbcL + ITS2* in our study resulted in 95% species resolution of barcodes recovered from herbal products, which is much higher than previous studies that used *rbcL + matK* (42% in Wallace *et al.*[3]; 66% in Stoeckle *et al.*[1]). DNA success rate was high in our study (91%) and in that of Stoeckle *et al.*[1] where they recovered barcodes from 90% of commercial herbal tea products. DNA barcode success rate was relatively low (48%) in the study by Wallace *et al.*[3]. This may be attributed to different manufacturing protocols, the type of plant material (for example, leaf, stem, roots and so on) used in the herbal preparation, or insufficient laboratory protocols used to extract, amplify and sequence haplotypes from herbal products. Herbal products contain plant secondary metabolites that may prevent barcode success. Herbal extracts contain complicated mixtures of organic chemicals (for example, fatty acids, sterols, alkaloids, flavonoids, glycosides, saponins, tannins and terpenes) that often result in PCR inhibition [53]. In addition, degradation at primer binding sites may also contribute to differential amplification success of selected genes in samples with potentially degraded DNA. In the Baker *et al.*[2] study, four dietary supplements could not be identified using the laboratory?s PCR amplification protocol, presumably because the DNA was degraded, possibly when heat was applied during the manufacturing process. Amplification failure in some samples, especially in *rbcL* gene, can be explained by the fact that primer sets used in this analysis may not be suitable for amplification of all species; we are developing new primer sets for mini-*rbcL* barcodes that will be easier to recover from degraded samples such as herbal products. The ideal protocol for barcoding herbal products will be realized as we build a more complete SRM herbal barcode library and continue to test more commercial products in the marketplace. Our study and others have documented that DNA can be routinely extracted from common forms of herbal dietary supplement extracts and powders, supporting a continued effort to explore DNA-based methods for quality assurance and quality control of herbal dietary supplements [1-3,54].

Many herbal products contain mixtures, which are particularly difficult to barcode. This difficulty is due to varied PCR success of selected genes in samples with potentially degraded DNA due to varied gene copy number and PCR bias; the chemical and physical properties of each piece of DNA can selectively amplify certain sequences more than others [55]. Several approaches could be developed for testing herbal mixtures such as real-time multiplex PCR and the use of next-generation sequencing [56]. In our study we chose to test only single ingredient herbal products. However, some of these products could contain more species than what was labeled. In order to search for other possible DNA barcodes we extracted multiple barcodes per sample in an attempt to obtain the most accurate estimate of identity within a sample. This included building barcode sample by species curves to see how many times we needed to sample to get an accurate estimate of species in a sample. Although we arrived at a figure of five to ten samples, we are currently using other molecular methods to verify the number of barcodes recovered from all of our herbal products that will overcome PCR bias and provide appropriate methods for testing herbal mixtures. Recent innovative approaches have combined morphological, molecular, and chemical techniques in order to identify the plant and chemical composition of some previous-generation smart drugs [57]. Such a multidisciplinary approach is proposed as a method for the identification of herbal blends of uncertain composition, which are widely available and represent a serious hazard to public health [57].

## Conclusions

Currently there are no standards for authentication of herbal products. Although there is considerable evidence of the health benefits of herbal medicine [53,58-66], the industry suffers from unethical activities by some of the manufacturers, which includes false advertising, product substitution, contamination and use of fillers. This practice constitutes not only food fraud, but according to the WHO, serious health risks for consumers [67]. A study of health claims made by herbal product manufacturers on the internet found that 55% of manufacturers illegally claimed to treat, prevent, diagnose or cure specific diseases [68]. Regulators such as the FDA and Canadian Food Inspection Agency (CFIA) may not have the resources to adequately monitor the dietary supplement manufacturers and their advertising claims, and there are concerns that the current regulatory system is not effective in protecting consumers from the risks associated with certain herbal products [69,70]. Chemical research studies have documented poor quality control and high content variability of active ingredients among products from a variety of manufacturers of herbal supplements [71,72]. This is partly because herbs contain complicated mixtures of organic chemicals, the levels of which may vary substantially depending upon many factors related to the growth, production and processing of each specific herbal product [73]. Although many manufacturers provide products with consistent levels of active ingredients through a process known as chemical standardization, this technique has uncertain effects on the safety and efficacy of the final product [71,74,75]. Many of the dangers of commercial plant medicine have been brought to light by DNA technology based studies that have identified contamination of herbal products with poisonous plants [70]. Eroding consumer confidence is driving the demand for a product authentication service that utilizes molecular biotechnology. One approach to vetting herbal product substitution and contamination is product authentication using DNA barcoding. Research studies such as ours and others [1-3] reinforce the importance of using DNA barcoding in the authentication of socioeconomically important herbal species [18]. We suggest that the herbal industry should voluntarily embrace DNA barcoding for authenticating herbal products through testing of raw materials used in manufacturing products, which would support sovereign business interests and protect consumers. This would be a minor cost to industry with a limited amount of bulk product testing, which would certify a high quality, authentic product. If the herb is known to have health benefits and it is in the product, then this would provide a measure of quality assurance in addition to consistent levels of active ingredients. Currently we are building an SRM DNA barcode library for commercial herbal species and standard testing procedures that could be integrated into cost effective 'best practices? in the manufacturing of herbal products. This would provide industry with a competitive advantage as they could advertise that they produce an authentic, high quality product, which has been tested using DNA-based species identification biotechnology, therefore gaining consumer confidence and preference. This approach would support the need to address considerable health risks to consumers who expect to have access to high quality herbal products that promote good health.

## Competing interests

The authors declare that they have no competing interests.

## Authors? contributions

SGN, SR and DS conceived of and designed the study, and carried out wet lab analysis and writing of the manuscript. MG carried out the fieldwork and contributed to the study design and writing of manuscript. SGN, SR and RS contributed to final editing and submission of the final manuscript. All authors read and approved the final manuscript.

## Supplementary Material

Additional file 1: Table S1 Standard reference material (SRM) herbal Barcode of Life Database (BOLD) accession numbers. Click here for file

Additional file 2: Table S2 List of GenBank accession numbers. Click here for file
